# A Secure Framework toward IoMT-Assisted Data Collection, Modeling, and Classification for Intelligent Dermatology Healthcare Services

**DOI:** 10.1155/2022/6805460

**Published:** 2022-06-29

**Authors:** Md Khairul Islam, Chetna Kaushal, Md Al Amin, Abeer D. Algarni, Nazik Alturki, Naglaa F. Soliman, Romany F. Mansour

**Affiliations:** ^1^Department of Information & Communication Technology, Islamic University, Kushtia 7003, Bangladesh; ^2^Chitkara University Institute of Engineering and Technology, Chitkara University, Rajpura, Punjab, India; ^3^Department of Computer Science & Engineering, Prime University, Dhaka 1216, Bangladesh; ^4^Department of Information Technology, College of Computer and Information Sciences, Princess Nourah bint Abdulrahman University, P.O. Box 84428, Riyadh 11671, Saudi Arabia; ^5^Department of Information Systems, College of Computer and Information Sciences, Princess Nourah Bint Abdulrahman University, P.O. Box 84428, Riyadh 11671, Saudi Arabia; ^6^Department of Mathematics, Faculty of Science, New Valley University, El-Kharga 72511, Egypt

## Abstract

The abnormal growth of the skin cells is known as skin cancer. It is one of the main problems in the dermatology area. Skin lesions or malignancies have been a source of worry for many individuals in recent years. Irrespective of the skin tone, there exist three major classes of skin lesions, i.e., basal cell carcinoma, squamous cell carcinoma, and melanoma. The early diagnosis of these lesions is equally important for human life. In the proposed work, a secure IoMT-Assisted framework is introduced that can help the patients to do the initial screening of skin lesions remotely. The initially proposed approach uses an IoMT-based data collection device which is accessible by patients to capture skin lesions images. Next, the captured skin sample is encrypted and sent to the collected image toward cloud storage. Later, the received sample image is classified into appropriate class labels using an ensemble classifier. In the proposed framework, four CNN models were ensemble i.e., VGG-16, DenseNet-201, Inception-V3, and Efficient-B7. The framework has experimented with the “HAM10000” dataset having 7 different kinds of skin lesions data. Although DenseNet-201 performed well, the ensemble model provides the highest accuracy with 87.22 percent as well as its test loss/error is lower than others with 0.4131. Moreover, the ensemble model's classification ability is much higher with an AUC score of 0.9745. Moreover, A recommendation team has been assigned to assess the sample of the patient as well as suggest the patient according to classified results by the CAD.

## 1. Introduction

In healthcare, the integration of medical hardware devices, smart systems, and apps with cloud storage and computing by using the Internet connection is referred to as the Internet of Medical Things (IoMT) [1]. After the IoT was introduced, it drastically reduced the number of unnecessary hospital visits by connecting patients to their doctors and allowed medical data to be sent over a secure network from anywhere. It not only saves time and effort but also shows how important it is to come up with cost-effective solutions [2]. The usage of IoMT in the community assured that data is shared securely and privately across the network, and it can be accessed remotely by patients and diagnostic centers at any time and from any location [3].

IoMT-assisted approaches provide substantial breakthroughs in a variety of medical sectors that demand careful investigation, monitoring, and early diagnoses, such as cervical cancer [4], diabetes [5], heart disease [6], breast cancer [7], ophthalmology [8], and infectious diseases [9] which are diagnosed at an early stage as well as monitored using IoT-based medical technology. In dermatology, it is important to identify skin lesions (nonmelanoma) in the early stages of their development to avoid further complications such as melanoma [10]. American citizens are at risk of developing skin cancer than others. Skin cancer affects one out of every five Americans, and one person dies from it every hour [11].

A skin lesion is a condition that is different from normal skin. In another way, it can be described as an abnormal change of the skin compared to the surrounding tissue. The American Society defines a skin lesion as an abnormal lump, bump, ulcer, sore, or colored area of the skin [12]. Skin lesions are a risk factor for skin cancer, and they progress slowly toward the development of malignant cells. For instance, they were closely linked to an increased risk of basal and squamous cell carcinoma [13]. However, skin cancer prevention would be possible if early detection of various skin lesions were possible in any case [14]. In this study, seven skin lesions are described and detected including dermatofibroma, vascular lesions, actinic keratoses, benign keratosis-like lesions, melanocytic nevi, melanoma, and basal cell carcinoma.

Benign keratosis-like lesions include seborrheic keratosis and lichen-planus-like keratoses (LPLK). Seborrheic keratosis (SK) is a benign skin tumor that develops from cells and is found across the external surface of the skin. It is a noncancerous skin lesion/growth that does not develop skin-related cancer. According to a study in 2022, SK is common among older people and 89% of older people had been diagnosed with this lesion in brazil. However, 24% of younger people had at least one SK lesion [15]. Similarly, LPLK is prevalent in older adults as a result of an inflammatory response or immune system failure that damages the skin inadvertently [16]. On the other hand, actinic keratoses (AK), alternatively referred to as solar keratoses, sun spots, or precancerous spots, are premalignant squamous lesions [17] and have the potential of developing cancer lately [18]. One in every 60 Americans over the age of 40 seems to have AK lesions, making it the 3rd most common skin disease in the USA [19]. Vascular lesions are a type of skin and basement membrane anomaly that can occur during or shortly after birth. Therefore, the treatment of acquired vascular birthmarks is one of the most frequently requested and performed cutaneous laser procedures [20]. Dermatofibromas are benign fibrous nodules that are formed when extra cells accumulate in the deeper layers of the skin and are predominantly found in the tissues including its lower legs [21]. Dactylofibromas were found in nearly three percent of skin biopsy samples taken at the diagnostic laboratory [22]. Basal Cell Carcinoma (BCC) is a skin cancer that grows on the skin's surface, and it is the most prevalent form of skin cancer and perhaps the most common type of cancer in general [23]. Because of the low mortality rate associated with BCC, the incidence records are not reliable and up-to-date. However, the rate of BCC in Europe has risen to 5% in the last few years, but only 2% in the United States; an estimated 4.3 million instances occur annually in the United States [24]. Melanocytic nevus is a type of melanocytic tumor that develops in the cells of nevus where it acts as a precursor to cutaneous melanoma and indicates an increased chance of acquiring cancer [25]. Melanocytic nevus that occurs in newborns and is present in the head and neck is known as a congenital melanocytic nevus. Congenital melanocytic nevi affect 0.2 to 6 percent of newborns around the world [26]. It usually begins on the skin, but it may also affect the mouth, intestines, and eyes. Literature review indicates that the overall number of instances of nonmelanoma skin cancer is 1,042,056, and melanoma skin cancer is 287,723 [27]. These statistics surely show the risk of being diagnosed with melanoma.

The biopsy technique is widely used in almost every medical lab to diagnose skin cancer. A biopsy is a treatment modality in which a small amount of tissue is removed and observed under the microscope. If an initial examination reveals that an area of the body's tissue is irregular, a doctor should suggest a biopsy [28]. There are various types of biopsy techniques such as punch, shave, incisional, and excisional biopsy [29]. A punch biopsy is a form of biopsy used to diagnose or heal skin cancer such as BCC. Punch biopsy has almost 81% diagnostic accuracy for BCC [30]. It is the most common biopsy procedure, and it involves cutting a cylindrical specimen of skin tissue with a circular blade [31]. However, punch and shave biopsy cannot examine deep tissue whereas shave biopsy is widely used for nonmelanoma skin lesions like seborrheic keratosis. In cases of probable melanoma, an excisional biopsy is frequently employed to evaluate deeper tissues of the afflicted skin [28, 32]. Several complications may occur during biopsy to diagnose skin cancer, such as pain, bleeding, damage to other tissues, infection, incorrect biopsy site, or difficulty covering the biopsy area, as well as other factors such as taking more time, going to the operating room, and costing for biopsy [28, 33]. Even an attack can occur during a biopsy which is known as a vasovagal attack. The most obvious type of syncope is vasovagal syncope, which occurs most often in anxious patients as well as those with an abnormal autonomic nervous system [33].

The complication of biopsy paves the way for alternative approaches to diagnosing skin lesions and cancer [34]. Although the dermoscopy methodology was invented in the seventeenth century, it has gained popularity recently due to its noninvasive examination method [35]. In recent years, Deep learning and segmentation-based algorithms have been utilized to detect and categorize skin lesions and cancer [36]. This technology ensures high precision while also saving time and money [37]. Therefore, early detection and remote monitoring are possible due to technological advancements such as IoT, smartphones, computer-aided diagnosing using deep neural networks, and cloud computing. Hence, the main contributions of the proposed work are as follows:

- An IoMT-Assisted Framework is proposed for remote data collection and processing.
- A secure encrypt/decrypt data transmission model is proposed for cloud storage.
- A data-driven approach is developed using ensemble deep learning models to classify skin lesions from skin images of patients.
- A proposed framework is examined with a benchmark dataset having seven classes of skin lesions.
- The proposed model is validated on collected skin images at home by various patients using smart devices like mobile and tablets.

The rest of the paper is organized as follows.  Section 2 highlights the state-of-the-art toward the problem domain. The description of the proposed methodology is presented in Section 3.  Section 4 describes the evaluation metrics employed with their experimental results and analysis. The details of the discussion on achieved results are presented in Section 5. Later, in Section 6, the whole work is concluded with future scope.

## 2. Related Work

Deep/machine learning is an emerging technology to automate our day-to-day life tasks and reduce time and cost. They have been widely used in various fields like home/office, agriculture, industry, and healthcare [38]. But, in the medical sector, its implantation is increasing nowadays including medical imaging. Medical imaging is implemented in different image processing or diagnosing techniques like MRI, X-ray, ultrasound, endoscopy, electrocardiography, etc. In medical imaging, computer vision technology techniques are highly used to classify various types/targets [39].

One of the most essential aspects of automation in the present day is the collection of data from various sources. People go to diagnostic centers to examine their health issues, which is both time-consuming and expensive for them. So, the researcher came up with IoT-based data collection so that they could figure out what was wrong without any assistance at home. IoT is implemented in power systems and energy-efficient smart buildings for data collection [40, 41]. In the medical field, it is a new concept with no clear explanation of how it works. Privacy protector, on the other hand, uses a hidden sharing method called SW-SSS to collect and transmit data [42]. Secure data, a data collection system, has been introduced with proper security in the cloud computing layer. The layer employed a database distribution mechanism in order to ensure the security of patient data stored in cloud storage [43]. IoT-induced data collection and monitoring for immediate medical treatment were proposed by Xu et al. [44]. While the studies described the data collection system's workflow, the system's design and implementation remain unclear. Furthermore, they failed to properly specify the IoT devices and sensors used in their research. In this work, we have tried to cover these gaps, and part of our work is available as a preprint [45].

Shen et al. [46] presented a study of medical image processing such as classification, pattern recognition, and segmentation using deep neural networks in the contemporary medical arena. They specify several state-of-the-art methods for carrying out the job. In addition, certain disadvantages are mentioned, such as data limitation, enhanced feature extraction and representation techniques for better precision, or black box-like character of deep learning methods. In [47], the application of deep learning approaches in the various health sectors (medical imaging) demonstrated such as histological/microscopic elements identification, gastrointestinal early diagnosis, cardiac/tumor detection, and Alzheimer/Parkinson detection are explored. They looked at a number of studies that used either pretrained (GoogLeNet, Alex Net, and LeNet) or personalized deep learning models to detect. They also defined various datasets that are often used to train a reliable and accurate model for a particular health problem. Using machine learning techniques, Khan and Algarni [6] updated an IoMT (Internet of Medical Things) for heart disease diagnosis. To increase the accuracy of the prediction, they used self-swarm optimization and an adaptive neurofuzzy inference method. They assessed the risk of heart disease by using data on chest pain, cholesterol levels, blood pressure, sex, age, and blood sugar levels. In [48], the “Wisconsin Diagnostic Breast Cancer” dataset and machine learning algorithm has been employed to detect breast cancer. In one of our studies, we have deployed deep learning as well as machine learning algorithms to identify the existence of diabetes at an early stage [5]. They did not, however, described how the IoMT device helped/linked to their proposed machine learning approaches.

In case of skin lesions classification, 20 dermatologists and a Faster Region-based CNN (FRCNN) model are compared (malignant and benign tumors), where FRCNN has outperformed accredited dermatologists. However, they did not use any other pretrained models or fine-tuning to increase accuracy [49]. Another study by Li and Shen [50] classified skin lesions as melanoma using deep learning methods. They used a fully connected residual network for segmentation and classification. Further lesion index calculation unit has been used to validate the result of the classification. In their approaches, no pretrained weight value was used to increase the accuracy. Besides, they used only the shifting procedure for data augmentation. In [51], the authors used image enhancement techniques and segmentation techniques and then extracted 15 features from each image which they fed to the deep neural network and hybrid AdaBoost-SVM model. They did not employ any data augmentation techniques. VGG-16 is used to train the skin melanoma detector classifier [52]. They used random weight initialization for training and fine-tuning on the VGG-16 network to improve accuracy. But no experiments about fine-tuning the different layers have been carried out and their accuracy metric is very low compared to the recent study. Masood et al. [53] discussed IoT-based computer-assisted pulmonary cancer detection systems which gather data using wearable sensors and classification of computed tomography images found from online sources to evaluate cancer stage. They did not propose any automated device to capture CT images from patients.

IoMT is an integration of sensors and software to automate our daily life by collecting, managing, and transmitting data over a network. In [54], an E-health monitoring system is created that tracks a person's life cycle and links them to a health management service provider. Their IoMT device is used for tracking diabetes, pulse rate, kidney function, etc. However, they failed to mention the IoMT device that would be used to test their hypothesis. Pinto et al. [55] employed a healthcare system for aging people to assist them with regular monitoring. They developed an android app called “We-Care” with a secure gateway that gets information from the “We-Watch” wristband. But they did not mention a proper description of what types of data will be collected and also no specific task of the app has been mentioned. Recent developments pave the establishment of a skin care and monitoring device called SkinAid, an IoMT pipeline, for skin lesions, which incorporates GAN-based data augmentation [56]. Similarly, numerous IoMT devices for skin lesions classification approaches have been developed without a clear explanation of how the device might be used in a home setting [57, 58].

A massive amount of data is created by IoT devices in health care and it is critical to manage the vast amounts of data by IoT itself due to its low storage and computation power. To address the issue, numerous approaches are being used, including cloud computing on cloud servers [59]. Additionally, cloud-based Internet of Things devices enable clinicians to remotely view patient data [60]. A pipeline was established with the integration of IoT and cloud computing in order to give e-healthcare to diabetic patients [61]. An IoMT-based device created by Kodali et al. [62] was used to collect medical information and archive it in the cloud for further assessment. Cloud-fog computing was employed to address the data availability to the IoMT-based healthcare by Mahmud et al. [63]. The fog cloud aids in cost reduction and easy to ease data accessibility toward the monitoring body as well as it can ensure security by using various algorithms and cipher technologies [42, 43].

## 3. Proposed Methodology

This section illustrates a data collection system based on IoMT and describes a method for detecting skin cancer using a deep neural network.  Figure 1 represents our proposed methodology for a better understanding of our hypothesis.

First of all, the image of the infected skins is captured by the Raspberry Pi Camera which is integrated into a Raspberry Pi board. After obtaining an image of the patient's affected skin, two significant steps are taken to transfer the data to a central repository, namely, the installation of an operating system and the configuration of the Internet facility.

The collected image is subsequently sent to a CAD (Computer-Assisted Diagnosis) system for analysis. CAD system preprocess the image for further processing. Then, an image segmentation technique is used to separate the target object from the image, and the feature extraction technique is then extended to the segmented area of interest. Further, the data is separated into train, validation, and test sets. At last, the classifier model is used to identify each patient's current condition. The output of the classifier is transferred to the central repository where the recommendation team will further assess the outcomes. They will notify the patients regarding his/her current conditions and will be recommended by the recommendation body. And the collected data and output will be stored in the cloud storage for future model training and assessment. This helps to make our infrastructure more stable in the future.

### 3.1. Patient Connection with the Smart Healthcare

A patient is the beneficiary of all medical services rendered by health providers. In this study, the patients are monitored to identify the existence of skin cancer using modern technology (IoMT and deep learning) without the involvement of pathologists. Therefore, the patient can easily utilize the IoMT-based device, which is connected to the CAD system, to evaluate the skin lesions condition and prescribe accordingly at any time without going to the hospital.

### 3.2. IoMT-Based Data Collection System for Skin Lesions

The Internet of Things corresponds to a collection of interconnected devices that can capture and transmit data over a mobile or wifi network without human interference. IoMT allows objects to be controlled accurately from a remote area with the help of network infrastructure and computer-assisted systems. In the future, it will be utilized for a new and significant purpose that will traverse borders and even the entire planet and frequently incorporate into a variety of fields and gadgets in order to work in a variety of domains [64]. In our IoMT-based data collection system, a Raspberry Pi 4 Model B has been incorporated that has 8 GB RAM in it, as shown in Figure 2 [65]. The board incorporates the Raspberry Pi Camera Module 2 (8 MP) chipset with flash module version V2, which is a small and portable camera that supports the Raspberry Pi via the serial protocol Mobile Industry Processor Interface (MIPI) [66]. It is now feasible to use multiple lenses that can automatically change the focus and exposure as well as mount stable video. This camera is used in deep learning, machine learning-based projects such as recognition, classification, and other functions [67]. During the COVID-19 pandemic situation, it was difficult to handle a large number of people who are probably infected by the virus. To assess the patient's status, such as fever and cyanosis, a Raspberry Pi board and camera-based IoMT device was constructed [68]. An Internet-free Computer-Aided Diagnosis (CAD) system for evaluating skin lesions was built using a Raspberry Pi3B+ and a camera [69].

In our framework, a 3.5-inch UCTRONICS touch screen connected with the Pi board displayed the collected data sample and process the data using various applications. In our proposed method, we have introduced Linux operating system in order to set up essential software which will assist in transmitting the images to the cloud storage. Moreover, we also need battery backup as well as a storage facility for the data. Thus, a standard V3 battery backup is included as well as a 16 GB SD card for the memory facility. The user will utilize the Linux environment to run the applications necessary to assess their skin condition.

### 3.3. Computer-Assisted Diagnosis (CAD)

The notion of CAD began to evolve slowly after the invention of the modern computer in the late 1950s. Another milestone was reached in 1960 with the first successful computer-aided medical image analysis (CAMI) [70]. However, it was created only for the purpose of studying its future prospects. It was mostly utilized in medicine for analysis and decision-making. Swender et al. [71] built the first effective Computer-Aided Diagnosis (CAD) system, which made use of patient records from hospitals. In Figure 3, we have demonstrated the flow diagram of our proposed CAD. This CAD will incorporate all the procedures to classify skin lesions using deep learning-based approaches.

#### 3.3.1. Collection of Dataset

Data collection is the most critical step in this study. Without a large volume of data and careful identification of each data point, it is very difficult to collect information and learn more. We have therefore suggested an IoMT base stable, sensible, and simple Pi camera for our data collection method in our study. Although we initially train our classifiers with a publicly accessible dataset. There are many publicly available datasets, like “BCN20000” which consists of almost 194 k dermoscopic images collected from Barcelona's hospital from 2010 to 2016 [72]. “Human Against Machine with 10000 training images (HAM10000)” consisted of almost 10015 images of dermatoscopic skin lesions tagged with the correct labeling by a pathologist or multistep follow-up, expert opinion, or in vivo confocal microscopy validation [73]. “PAD-UFES-20” is a comparatively new dataset composed in 2020 of almost 2298 images from 1373 using smartphones [74]. Fitzpatrick Dataset has been developed by Groh et al. [75] that includes almost 17 k clinical images for classifying 114 different skin lesions or cancers. MED-NODE dataset contains 170 images only whereas 70 melanoma cases and 100 nevus cases [76]. Edinburgh skin lesions dataset includes 1.3 k images of 10 lesions [77]. Wen et al. [78] represented skin lesions related to 21 datasets (containing 1000 k images) and atlases that also included age, sex, region, ethnicity, and other factors.

#### 3.3.2. Image Prepossessing

The captured image has to be preprocessed before feeding the image into the neural network so that the neural network can filter further information in each layer. Traditional methods for image preprocessing refer to the transformation of images into raw data that can be fed by the neural network. The aim of preprocessing is to optimize image data that eliminates unwilling information or improves those image features that are necessary for further pattern identification [79]. In one respect, choosing the very first set of pixels in an image in the RGB color space is a procedure performed by different algorithms operating on a computer device [80]. Techniques such as resize, mean normalization, standardization, smoothening, and blurring are used in image preprocessing. The HAM10000 images are resized to 64 *∗* 64 and 96 *∗* 96 in the RGB color space. We also conducted a data augmentation technique to supply the neural network with a wide variety of images as a batch. Data augmentation includes rotation, scaling, shift, and fill mode [81].

#### 3.3.3. Feature Extraction

The patterns of the object in an image are referred to as features. A triangle, for example, has three corners and three sides, which are the characteristics that our eyes use to recognize the triangle. Similarly, the convolutional network can remove key features from each image to aid in the identification of a certain class or target value. Convolutional kernels remove valuable features from the original image, reducing the dimension and resulting in more efficient features with fewer redundant data. This method is known as a feature mapping process. This reduced representation of the original image would provide a detailed understanding and more accuracy [82]. More specifically, each hidden layer will extract important features and feed them into the next layer for further feature extraction. Moreover, they not only extract features but also identify the interactions among the extracted features. And the last hidden layer will produce the final features and interactions for the output layer [83, 84]. The output layer used the Softmax classifiers in order to classify the skin lesions.

#### 3.3.4. Classifier

A classifier is an algorithm that converts data into one of several categories or classes. And convolutional neural network or ConvNet is one type of neural network mostly used in image classification. There are several layers in the convolutional neural network, such as the input layer, hidden layer, and output layer. Each layer has several neurons or nodes that take information from the previously hidden layer or input layer that used the mapping function to process the data and transfer it to the next layer [85, 86]. One of the categories is generated by the output layer. The input layer takes raw data, which in our case would be the tensor of the original image. And this overall mechanism is supervised learning because the computer trains using the target value of the training dataset [87].

*(1) Convolutional Layer*. The convolution layer is used to extract information/features using kernel/filters. Kernel size is smaller than the input image which scans the image's spatial position step by step. Then, bias and other required elements are added, and also weighted sum is calculated. At last, the output of the layer is passing through the nonlinear activation function to get new features for the next convolutional layer [85, 88]. Generally used activation functions are ReLU, sigmoid, tanh, etc. The function is processed in a convolutional layer denoted by

(1) $$\begin{array}{c} x_{j}^{l}=f\left(\overset{m}{\underset{i}{\sum }}\left(x_{i}^{l-1}{\;}^{*}w_{ij}^{l}+b_{j}\right)|.\right. \end{array}$$

*x*_*j*_^*l*^ denotes the *j*^th^ features of *l*^th^ layer where *w*_*ij*_ is the weight between the *j*^th^ feature of *l*^th^ and *i*^th^ feature of *l* − 1^th^ feature. And *b*_*j*_ is the bias of *j*^th^, and *m* is the number of features created in *l*^th^ layer.

Traditionally, convolutional layer kernel size is 3 *∗* 3. It derives the most important features and less information loss occurred. Besides, it reduces the number of parameters and hence reduces the time of calculation. Furthermore, kernel sizes 3 and 5 performed well when combined with a large number of hidden layers [89].

*(2) Pooling Layer*. The pooling layer is generally used between two convolutional layers. It tries to compress the features found from the previous convolutional layer. Compression is done by taking the max or average value from a particular region. Max pooling is mostly used as it produces the best result [85].

*(3) Fully Connected Layer*. The convolutional and pooling layers provide room for the features of the images. Fully connected layers are layers where all the previous layer neurons are connected to the next layer. It can be considered an affordable way to learn a linear function from the feature region [90].

*(4) Output Layer*. The Softmax classifier is typically employed as an output layer for multiple-class classification. Suppose that there are *J* images, where each image is labeled with a value *y*_*i*_ ∈ (1,2,3,…, *k*) whereas *k* is the total number of classes in the dataset and *y*_*i*_ denotes the targeted label. For each image *x*_*i*_, there will be *k* probability score corresponding to each class. So, the equation is

(2) $$\begin{array}{c} h_{\theta }\left(x_{i}\right)=\left[\begin{array}{c} p\left(y_{i}=1|x_{i};\theta \right)\\ p\left(y_{i}=2|x_{i};\theta \right)\\ p\left(y_{i}=3|x_{i};\theta \right)\\ \ldots \ldots \ldots \ldots \ldots \ldots ..\\ \ldots \ldots \ldots \ldots \ldots \ldots ..\\ \ldots \ldots \ldots \ldots \ldots \ldots ..\\ p\left(y_{i}=k|x_{i};\theta \right) \end{array}\right]. \end{array}$$

In (2), the sum of all the classes' probability is equal to 1 and *θ* represents the parameter of the classifier (Softmax classifier).

There are several ConvNet classifiers in deep learning, e.g., Xception, VGG-16, ResNet50. ResNet101, DensNet121, MobileNet, and so on.

*VGG-16*. The VGG-16 architecture is a convolutional neural network, and it was used in 2014 in an annual competition called the “ImageNet Large Scale Visual Recognition Challenge.” The ImageNet dataset includes RGB-channel images with a fixed size of 224 *∗* 224; in our case, it is 96 *∗* 96. In this architecture, 16 layers are used, including convolution layers of a 3 × 3 filter with stride 1 and always the same padding and max pool layer of a 2 × 2 filter with stride 2 [91].
*DenseNet-201*. One of the neural networks for visual object recognition is DenseNet-201, which has 201 layers. The network's image input size is 224 *∗* 224 pixels. The name DenseNet arises from the fact that each layer in a DenseNet architecture is linked to every other layer. Instead of using summation, the DenseNet paper suggests concatenating outputs from previous layers. Transition layers are used by DenseNet. Convolution with a kernel size of 1 is accompanied by 2 × 2 average pooling with a stride of 2 [91].
*Inception-V3*. Inception-v3 is a convolutional neural network architecture from Google's Inception family V3. The third version in a series of Deep Learning Convolutional Architectures makes many improvements, such as Label Smoothing and Factorized 7 × 7 convolutions. It was trained using a dataset of 1,000 classes from the original ImageNet dataset, which was trained with over 1 million trajectories [91].
*Efficient-B7*. EfficientNet-B7 achieves new state-of-the-art 84.4 percent top-1/97.1 percent top-5 accuracy despite being 8.4% smaller than the best current CNN by scaling up the baseline network. The total number of layers in EfficientNet-B7 is 813, and all of these layers can be created using only five modules. Module 1 serves as a starting point for the subblocks, module 2 serves as a starting point for the first subblock of each of the seven main blocks except the first, module 3 serves as a skip link for all of the subblocks, and module 4 helps to combine the skip connections in the first subblocks. Finally, module 5 connects each subblock to the one before it in a skip link, and this module is used to merge them [91].
*Ensemble Model*. An ensemble model is a single model where multiple model's (in our case IceptionV3, VGG-16, DensNet-121, Efficient-B7, and a custom model) predictions are combined together and predict one single outcome. It is like a decision-making board that decides based on the predictions of different models [92]. Generally, a base model has a unique error on dataset samples, but the ensemble model uses all the model's predictions which reduce the error more than a base model. Different machine and deep learning-based studies used the ensemble model for better accuracy and to get a robust model for classification tasks [92–94]. In our case, we have used averaging ensemble model as shown in Figure 4. In an averaging ensemble model, we take an average of all models' probability for classes and make a final decision based on the average outcome of each class [95]. Suppose that we have *L* models where each model *l*_*i*_ predicts *k* probability as we have *k* classes. Then, the final class of the ensemble model for a particular image *x*_*i*_ will be
  (3) $$\begin{array}{c} E\left(x_{i}\right)=\frac{\sum_{i}^{L}h_{\theta }^{l_{i}}\left(x_{i}\right)}{L}. \end{array}$$

In (3), *E*(*x*_*i*_) denotes the ensemble outcome for *x*_*i*_ image where *h*_*θ*_^*l*_*i*_^(*x*_*i*_) defines *i*_th_ ∈ *L* model's classifier function outcome.

### 3.4. Central Repository

The repository is a disk on which all of the data will be kept, including configuration information. In the central repository, we maintain our data in an uncompressed form for easy handling, accessing, and transmission of the data. The central repository is useable by a computing device via a communication network. Depending on the user's request, a communication network can be established with the central repository [96]. In our pipeline, we have included a cloud storage-based repository for storing and managing data linked to skin lesions. However, there are a few factors that must be considered in order to have an effective repository in the medical field, including accessibility, security, management, scalability, and regular maintenance. As a result, a cloud server is a feasible alternative; furthermore, it is both cost-effective and simple to transfer data to a remote location [97]. Despite the benefit, cloud storage has some limitations such as user limitations, storage crashes, or hacking [98]. So, we proposed multicloud facilities which provide data security in various storage, by replicating the data in different cloud servers, as well as parallel computing for user queries [99].

### 3.5. Recommendation System

The proposed smart healthcare stores the collected skin lesion images and the classified outcomes in a cloud repository for future justification. Then, the information will be forwarded to the medical recommendation team, who will provide suggestions for specific measures to be followed [100]. In developed nations, people are more worried about their physical and mental health. However, in less developed and developing countries, it is quite hard for them to keep track of their health on a regular basis. The planned smart healthcare may enable people to contact medical professionals even while they are at home, therefore making life easier and accessible to all the facilities [101].

The recommendation system can be divided into five steps/phases such as data collection and evaluation, information exchange, regular or emergency scheduling, remote monitoring, and cloud storage maintenance.

#### 3.5.1. Data Collection and Evaluation

The patient could collect skin samples using the IoMT-based data collection system and then submit the result to the cloud server for evaluation. The submitted data will be checked and confirmed by the recommendation team (RT) for further classification. The submitted sample can be rejected by the RT if the image is not perfectly captured by the patient as well as request for further sample submission.

#### 3.5.2. Information Exchange

After confirming the sample, the RT will further proceed with the data for classification by the CAD system installed in the cloud. The outcomes of the sample will be redirected toward the patient device with the required suggestions.

#### 3.5.3. Regular or Emergency Scheduling

According to the result, the patient could be requested for regular or emergency scheduling. In case of a medical emergency, the recommendation team will notify the doctor or pathologists to prepare for handling the emergency situation [102].

#### 3.5.4. Remote Monitoring

The prescribed patient will follow the required treatment such as regular diagnosing and medication. The recommendation team may use the patient's previous data from the central repository in order to compare the patient current status. The patient may need to be sent to a hospital for further examination or treatment if required [4].

#### 3.5.5. Cloud Storage Maintenance

Multicloud storage would have all the confidential data regarding the subscribed patient. So, regular maintenance of the cloud server is required. Moreover, there are issues related to such unauthorized access [103].

This entire operation benefits not just those in impoverished nations who face challenges in all aspects of life but also people from developed nations who want to save time [104].

## 4. Experiments and Results

This section describes the result of the proposed methods in our methodology and their experimental comparison.

### 4.1. Dataset Management and Data Visualization

HAM10000 is the selected dataset for our proposed methodology. We have split our dataset into a train (7210), test (1002), and validation (1803).

HAM10000 dataset has almost 10015 dermoscopic images of seven different skin lesion diseases.  Figure 5 shows the number and percentage of dermoscopic images regarding each skin lesion disease. And it is clearly noticeable that the dataset is imbalanced.

### 4.2. Experimental Setup

In the experimental setup, we have discussed the computational and structural configuration for our proposed methodology in detail. We have deployed python packages such as Numpy, Scikit-learn, Pandas, Keras, and TensorFlow. Keras is extensively used for neural network training with TensorFlow as a backend. The parameters and hyperparameters used in the training process are represented in Table 1 [105].

The dataset contains images of different sizes. So, we resized the images to a 96 *∗* 96 pixel size so that they can be easily fed to neural networks. Then, we converted the ground truth to categorical values. Our models are trained using the train and validation sets by learning the pattern of the classified images. The test set has been retained to assess our models' performance on unseen data. Different pretrained models, more specifically transfer learning, are introduced to get the best classification result out of the dataset. But the top classification layer (including flatten, fully connected layer, and softmax) is customized so that it will be well aligned with the data and get the best results out of it. ImageNets' weights are initialized as the initial variable of the neural network. Then, data augmentation techniques are used in each epoch before feeding to the neural network. The experiment used 50 epochs in the training phase, which implies that the entire dataset was processed through the DL algorithms 50 times. In each epoch, there are 144 steps for the training dataset and 36 steps for the validation dataset with a batch size of 50. Different optimizers have been used alternatively in various classification analyses like Adam, RMSprop, etc. In our case, we have used Adam as optimizers in all the selected deep learning models. “Categorical cross-entropy” is used as a loss function in the experiment. We also used the learning rate reduction function to reduce the learning rate as the epoch increases [106].

### 4.3. Evaluation Metric and Results

In this section, we have described the evaluation metrics used to validate the performance of the proposed methodology. In general, accuracy is used to define the performance of a particular model. But in medical imaging, the accuracy of the model is not enough to have an exact idea of the model. So, there are many more metrics to evaluate a deep learning model like precision, recall, ROC curve, and *F*1 score. We have used all of these metrics to evaluate and understand a model's performance.

The confusion matrix is considered the most comprehensive way to describe all the metrics and is determined by the following:

- True Positive-predicted target label true and ground label also true
- False Positive-predicted target label true but ground label actually negative
- True Negative-predicted target label negative and ground label also negative
- False Negative-predicted target label negative but ground label actually true

So, a target label correctly classified means that it should be True Positive (TP) or True Negative (TN). Similarly, when the target label is wrongly classified, it will be False Positive (FP) or False Negative (FN).

Accuracy is the sum of all correctly classified data points divided by all data points:

(4) $$\begin{array}{c} \text{Accuracy}=\frac{\sum \left(\text{True Positive}+\text{True Negative}\right)}{\sum \left(\text{True Positive}+\text{False Positive}+\text{True Negative}+\text{False Negative}\right)}. \end{array}$$

Precision defines the proportion of patients correctly predicted as having skin lesion/cancer against its predicted all lesion/cancer patients. That means the sum of all true positive labels is divided by the sum of all truly predicted labels and falsely predicted true labels, where recall/sensitivity specifies the proportion of patients correctly predicted as having skin lesions/cancer against actually all cancer patients. So, the sum of all true positive labels is divided by the sum of all actual true labels. They are determined by

(5) $$\begin{array}{c} \text{Precision}=\frac{\sum \text{True Positive}}{\sum \text{True Positive}+\text{False Positive}},\\ \text{Recall}=\frac{\sum \text{True Positive}}{\sum \text{True Positive}+\text{False Negative}}. \end{array}$$

Precision tries to minimize the false positive rates. So, in our case, with the increase of precision outlined that it is trying to reduce its wrongly predicted cancer patient. But recall is most important for our case. As we do not want to miss any cancer patients predicted as normal. Recall tries to minimize the false negative rates [107].

*F*1 score helps to understand both precision and recall from one score. We can take the average of both precision and recall, but it reduce the score drastically if any smaller (either precision or recall) value appear [108]. So, they come up with a balance equation which tries to more closer to the smaller value and give more accurate score that is:

(6) $$\begin{array}{c} f1-\text{score}=\frac{\sum \left(2\times \text{precision}\times \text{recall}\right)}{\sum \left(\text{precision}+\text{recall}\right)}. \end{array}$$

A function which we try to minimize or maximize is called objective function. However, when we sought to mitigate it precisely, we called it a cost function or a loss function. The cost function or loss function is used to describe all the good or bad points using a single scalar value. It helps to understand the error of a particular model and help to rank all the models. In our case we have used categorical cross-entropy. Categorical cross-entropy explicitly used for multiclass classification and described as:

(7) $$\begin{array}{c} \text{Categorical}-\text{cross}-\text{entropy}=-\sum_{i=1}^{\text{output size}}y_{i}\log\;{\overset{\wedge }{y}}_{i}. \end{array}$$

In our experiment, the dataset includes seven different skin lesions, which means the classifier performing multiclass classification as well as the dataset is imbalanced. Dermatofibroma, vascular lesions and actinic keratoses combined only 5.8% of the total dataset. Therefore, to better evaluate the classifier outcomes is not possible using ROC. Because ROC performed well for binary classification and balance datasets only. In the python environment, scikit-learn has introduced a new package to evaluate the multiclass classifier performance. It calculates AUCs for all the classes considering a particular class against all the other classes altogether. The ROC-AUC score allows an understanding of how well a classifier can be separated from different classifiers. Furthermore, the metric assist in analysing imbalance datasets more accurately compare to other metrics [109].

In Table 2, dataset's train and validation accuracy and train and validation loss for VGG-16, Inception-V3, Efficient-B7 and DenseNet-201 are shown.

Table 3 shows the testing data's accuracy, loss, precision, recall, F1 score and ROC-AUC score for all the deep learning models.

## 5. Discussion

In this research, we have proposed a framework for remote monitoring and diagnosis of skin lesions patients is shown in Figure 1. The patient has an IoT-based data collection device which he/she will use to collect dermoscopic images of the affected area (as shown in Figure 2). The device is also connected to a cloud storage so that the collected sample could be send over the network. Then the recommender team will further assess the sample for further processing such as the correct sampling and diagnosing using the Computer-Assisted Diagnosis (CAD) (as shown in Figure 3). The outcomes of the CAD classifier will be available for the patient as well as the recommender team. Moreover, the recommender team will suggest the patient for further self-care, medication or doctor appointment. In addition, the recommender team manages emergency situations by analysing hospital data from the cloud server.

We have introduced multicloud storage as the central repository. The multicloud provide parallel computing and security of the patient and hospital data in multiple server. Thus, if a crash occurs or an unauthorized user gains access, the recommender team will immediately disable the service. As a result, data on the other server is still safe for use. The proposed recommendation system is divided into five stage to cope up with any situation. It includes data collection and evaluation, information exchange, regular or emergency scheduling, remote monitoring and cloud storage maintenance.

In our study, we have established a Computer-Assisted Diagnosis (CAD) system which can detect skin diseases automatically using the image of skin lesions. First of all we have collected dermoscopic images from patient using IoMT device. In CAD we have then implemented a deep learning-based image classifier using transfer learning and ensembling of different models (as shown in Figure 4) for skin lesions classification. For transfer learning approach we have used popular pretrained models like VGG-16, Inception-V3, Efficient-B7 and DenseNet-201 etc. We have performed 50 epoch for each model on HAM10000 dataset. The final outcome of transfer learning is quite satisfactory.

Figure 6 depicts the relative positions of training and validation accuracy in each epoch for all four pretrained models, where Figure 7 shows the relative positions losses. In Table 2, show training and validation accuracy, loss etc. In Table 3 show the test's metrics, the visual representation of test accuracy and loss is shown in Figure 8.

The difference of VGG-16 model's train, validation and test accuracy is low, so the model neither overfit nor underfit. Inception-V3 test accuracy is comparatively low than other models. Both VGG-16 and Inception-V3 took less time to train in each epoch than the other two models. The test loss for Inception-V3 is higher than VGG-16.

Efficient-B7 took more times than other models because of its huge number of parameters to train. The model also shows a good accuracy (train = 91.82, validation = 85.14 and test = 82.93) with low loss (train = 0.2173, validation = 0.4829 and test = 0.6954). Efficient-B7's ROC-AUC score also good that means its separable/classification quality considerable. But DenseNet-201 has the best separable quality than any others model we have applied. DenseNet-201 have the best train (99.71%), validation (86.36%) and test (85.33%) accuracy. But its validation and test loss is higher among all the models.

In case of precision and recall, DenseNet-201 win the race with 85.32% and 85.32%, respectively. Precision defines the correctly predicted true positives (present of skin malignant) against total predicted true positives. Where recall/sensitivity defines the correctly predicted skin malignant against the total actual skin malignant cases.

Transfer learning took comparatively less time to train than baseline models. Because we have used preinitialized weights from “ImageNet.” ImageNet was trained on almost 14 million data for 20,000 classes [110]. So, it has a well established weights to train.

We also performed ensemble of our trained models. Ensemble model is like a decision-making board which reduce the generalisation error. In our case we have ensembled VGG-16, DenseNet-201, Inception-V3 and Efficient-B7 together using average ensembles methods. And our ensemble model is outperform than all other models on test dataset as shown in Figure 8. Not only loss is reduced to 0.41 but also accuracy is increased to 87.22% for test. Both loss and accuracy is improved than any other base pretrained models. The accuracy, recall, and *F1 score* of the ensemble model outperform than that of other models. Ensemble model's roc curve shown in Figure 8(c). In case of skin lesions classification, ROC-AUC score (with 0.9745) of ensemble model defines the best separable ability than any other models as far as we know.

In China, as of 2018 there are almost 12% of the population are older. Therefore, a smart-nursing pipeline proposed in order to remotely monitor them. However, Pinheiro et al. [111] did not describe about the tool required to develop the pipeline. Another study hypothesized a framework for skin lesions classification at home. But their work did not represent how the hardware are interconnected for the data collection system. Moreover, they did not specify how the smart diagnosing system managed such as recommendation team or automation [112]. Most of the smart diagnostic system for skin lesions did not propose a top-to-bottom pipeline for handling the issue [113–115]. However, Our proposed methodology is a top-to-bottom approach to handle the skin lesions remotely with proper suggestion from recommender team. The patient collect the data and send over network to the multicloud storage. The CAD system run the classifier to classify the skin lesions type and then pass the patients result to the central repository. A recommendar team have the access to the central repository. And they will prescribed or recommend the patients about next step. So, our IoMT and deep learning base Computer-Assisted Diagnosis (CAD) will help the patients to diagnosis skin diseases at home. It will reduce both the cost and time for diagnosis. This means that we have developed a comprehensive system for remote monitoring and diagnosis of skin lesions.

We do have some limitations in terms of our framework's long-term potential. For the patient, we did not propose a two-step authorization process. The facility is accessible to anyone who has the device. Moreover, Our long-term goal is to create a smartphone application that eliminates the need to buy a device. Furthermore, data transmission over the network is not encrypted. As a result, a skilled hacker could gain access to it.

## 6. Conclusion

In this research we have proposed an IoMT-based Computer-Assisted Diagnosis system in association with IoT-based data collection system. A deep learning model implemented in the CAD system which can classify skin lesions from skin images.

We have performed transfer learning models like VGG-16, Inception-V3, Efficient-B7 and DenseNet-201 etc. This models show exceptional performance for classifying skin lesions. Parameters tuning help us to increase our accuracy and produce more robust model on the dataset. We then ensemble all the models which outperform than any other models. Our deep learning method and pretrained models are available for more use of the classifier, as well as for researchers and students to help with more precise improvement.

Our IoMT-based CAD system is also connected to a central repository and a recommend team. A central repository is used to store data for further processing and use, and the recommend team assists a specific patient in learning about his or her current conditions and referring him or her to a specialist doctor. Overall, our IoMT-based CAD system connects the patient, diagnostic center, and doctor in a chain.

## Figures and Tables

**Figure 1:** Proposed methodology for IoMT-deep learning-based skin lesion classification and recommendation.

**Figure 2:** Our proposed IoMT-based data collection system which includes Raspberry Pi 4 Model B 3.5-inch touch screen, battery pack V3, memory card, Raspberry Pi Camera Module 2, and camera flash module V2.

**Figure 3:** Flow diagram of CAD which includes data collection, preprocessing, feature extraction and classifiers.

**Figure 4:** Flow diagram of average probabilities based on ensembling of various classifiers including VGG-16, Inception-V3, DenseNet-201, and Efficient-B7.

**Figure 5:** The HAM10000 dataset is divided into seven categories, each represented by a probabilistic paradigm in the pie chart.

**Figure 6:** Expression of accuracy in each epoch both for training and validation dataset. (a) DenseNet-201. (b) Efficient-B7. (c) Inception-V3. (d) VGG-16.

**Figure 7:** Expression of loss in each epoch both for training and validation dataset. (a) DenseNet-201. (b) Efficient-B7. (c) Inception-V3. (d) VGG-16.

**Figure 8:** Accuracy and loss on the test dataset of our trained model including ensemble model. (a) Test accuracy. (b) Test loss. (c) ROC curve.

**Table 1:** Hyperparameters utilized to train the deep learning models, as well as the parameters for data augmentation of the data.

	Value
*Data augmentation parameter*	
Rotation range	60
Width shift range	0.2
Height shift range	0.2
Shear range	0.2
Zoom range	0.2
Horizontal flip	True
Fill mode	Nearest

*Hyperparameter for DL models*	
Optimizer	Adam
Learning rate	0.0001
Learning rate reduction factor	0.5
Beta-1	0.9
Beta-2	0.999
Decay	0.0
Epsilon	None
Amsgrad	False
Input size	(96, 96, 3)
Output size	7
Number of epoch	50
Flatten layer activation function	ReLU and softmax
Shuffle	False
Batch size	64

**Table 2:** Train and validation metrics of deep learning models.

Model	Train accuracy	Train loss	Validation accuracy	Validation loss
VGG-16	92.74	0.1976	83.97	0.5837
Inception-V3	94.75	0.1444	83.58	0.6582
Efficient-B7	91.82	0.2173	85.14	0.4829
DenseNet-201	99.71	0.0086	86.36	0.8200
Ensemble model	—	—	89.36	0.3369

**Table 3:** Test metrics of deep learning models.

Model	Test accuracy	Test loss	Precision	Recall	*F*1 score	ROC-AUC score
VGG-16	83.33	0.7207	83.33	83.33	83.33	0.9074
Inception-V3	80.94	0.7858	80.93	80.93	80.93	0.9321
Efficient-B7	82.93	0.6954	82.93	82.93	82.93	0.9546
DenseNet-201	85.33	0.9501	85.32	85.32	85.32	0.9599
Ensemble model	87.22	0.4131	86.72	87.22	86.60	0.9745

## Data Availability

The data used to support the findings of this study are available at https://dataverse.harvard.edu/dataset.xhtml?persistentId=doi:10.7910/DVN/DBW86T
